The article "Variability in Platelet-Rich Plasma Preparations Used in Regenerative Medicine: A Comparative Analysis" was published in 2022. Journal: Stem Cells Int.

# Variability in Platelet-Rich Plasma Preparations Used in Regenerative Medicine: A Comparative Analysis

**DOI:** 10.1155/2022/3852898

**Published:** 2022-10-20

**Authors:** Raghvendra Vikram Tey, Pallavi Haldankar, Vivek R. Joshi, Rishi Raj, Ravindra Maradi

**Affiliations:** ^1^Department of Pathophysiology & Clinical Medicine, Western Atlantic University School of Medicine, Freeport, Grand Bahamas, Bahamas; ^2^Department of Biochemistry, Department of Interprofessional Chronic Care, Drexel University College of Medicine, Wyomissing, Reading, PA, USA; ^3^Department of Internal Medicine, Division of Endocrinology, Diabetes and Metabolism, Pikeville Medical Center, Pikeville, Kentucky, USA; ^4^Department of Biochemistry, Kasturba Medical College, Manipal, Manipal Academy of Higher Education, India

## Abstract

**Background:**

Platelet-rich plasma (PRP) and its derivatives are used in several aesthetic, dental, and musculoskeletal procedures. Their efficacy is primarily due to the release of various growth factors (GF), interleukins, cytokines, and white blood cells. However, the PRP preparation methods are highly variable, and studies lack consistency in reporting complete procedures to prepare PRP and characterize PRP and its derivatives. Also, all the tissue-specific (in vivo and in vitro) interactions and functional properties of the various derivatives/factors of the PRP have not been taken into consideration by any study so far. This creates a potential space for further standardization of the PRP preparation methods and customization of PRP/PRP derivatives targeted at tissue-specific/pathology specific requirements that would enable efficacious and widely acceptable usage of PRP as main therapy, rather than being used as adjuvant therapy. The main objective of our study was to investigate the variability in PRP preparation methods and to analyze their efficacy and reliability.

**Method:**

This study considered articles published in the last 5 years, highlighting the variability in their PRP preparation methods and characterization of PRP. Following the PRISMA protocol, we selected 13 articles for the study. The selected articles were assessed using NHLBI quality assessment tool.

**Results:**

We noted differences in (1) approaches to producing PRP, (2) extent of characterization of PRP, (3) small scale and large-scale preparation methods, (4) in vitro and in vivo studies.

**Conclusion:**

We identified two studies describing the procedures which are simple, reproducible, economical, provide a good yield of platelets, and therefore can be considered methods for further tissue-specific and pathology-specific standardizations of PRP and its derivatives. We recommend further randomized studies to understand the full therapeutic potential of the constituents of PRP and its derivatives.

The article "Variability in Platelet-Rich Plasma Preparations Used in Regenerative Medicine: A Comparative Analysis" was published in 2022. Journal: Stem Cells Int.

## 1. Introduction

It is evident now that autologous platelet-rich plasma (PRP) preparations have found several applications and their efficacy in some cases is well established. Most of the evidence is based on Class I/II clinical trials from around the world [1]. PPR is used widely in the field of aesthetic medicine and cosmetology as fillers or in rejuvenating procedures. In musculoskeletal injury, it is injected at the site of musculoskeletal and tendon injury showing promising structural and functionality improvements. PPR therapy is an approved and acknowledged procedure in dental treatment protocols. In wound healing studies, PRP injected into the nonhealing or chronic wound sites or its application in the form of dressing has shown appealing clinical outcomes [2]. The therapeutic effect of PRP is attributed to its ability to release distinct types of growth factors, cytokines, and interferons. They promote angiogenesis, fibroblast proliferation, epithelial cell proliferation, and healing at the site of the wound when used as an adjunct to standard wound care practice [3–5]. But unlike drugs/pharmaceuticals where the quality of a compound is ensured by a standardized mechanized procedure, the biologics field is in its adolescence. The protocols to prepare autologous PRP vary from one setup to another [1, 2]. This consequently adds variability to the outcomes of therapeutic procedures. The variability can be attributed to two main factors, PRP preparation procedure and patient-related factors [2, 5–9]. However, the preparatory procedures can be standardized, bringing them closer to the level of pharmaceuticals, to bring the product variability into an acceptable range. It is important to acknowledge the fact that like biologics, the approved pharmaceuticals also have variable outcomes, but they are favorable, backed with large volumes of scientific data and hence their acceptability as standardized treatment. The difference in the quality of PRP preparations arises from the fact that various setups tend to use variations of the same procedure to increase the quality of their PRP. The variations are seen in the amount of venous blood collected for processing, tubes used for collection, use of anticoagulant, centrifugation instruments, amount of G force used, time of centrifugation, temperature control, usage of additives/activators in PRP, pipetting methods (there is a human error involved here), the volume of PRP, storage methods, and duration of storage [2, 3, 9–11]. We have seen significant efforts in the direction of standardization of biologics, especially by the mechanization of the preparatory procedure using robotics and standardized kits. The effectiveness of the preparation procedure can be measured and compared if the PRP/PRP products are characterized, all the criteria transparently reported, and those characteristics are within an acceptable range. This is not always the case [1]. We have seen encouraging results in this aspect where recent studies have characterized PRP/PRP derived products across various criteria such as platelet number/platelet yield, amount of growth factors(GFs), proinflammatory cytokines, anti-inflammatory cytokines, immunophenotyping, platelet-derived extracellular vesicles, type and number of lymphocytes present, fibrinogen levels, prothrombin levels, P-selectin expression, IL-1ra levels, adhesion molecules, lysosomal enzymes, lipopolysaccharide (LPS) of platelet clot, and genes activated [2, 3, 11–16].

The article "Variability in Platelet-Rich Plasma Preparations Used in Regenerative Medicine: A Comparative Analysis" was published in 2022. Journal: Stem Cells Int.

The efficacy of the PRP preparation is measured in vitro using cell lines and in vivo studies. The subject/patient-related factors such as overall health and age also play a significant role when we think of the in vitro study outcome or the clinical outcome. The age-related variability has been seen in some factors but the overall quality of the harvest of PRP, when compared between perfectly healthy adults and elderly with comorbidities on medications, has been without statistically significant differences [5].

PRP is considered safe and natural because it is from an autologous source, prepared with minimal manipulation, with fewer risks of infection transmission, and no immune reactivity [17]. However, certain side effects have also been noted namely, injection site infection and injury to blood vessels and nerves, scar formation, calcification at the local site, allergic reaction to activated PRP, clot formation upon accidental intravenous injection, and soreness at the local site after an intramuscular injection has also been reported [17].

PRP has evolved over the generations. The first generation saw validation of concentrated platelets, growth factors (GFs), development of automated PRP preparation devices, and recognition of anticoagulant's role in sample collection. The second generation introduced modifications to preparation protocols and developments of novel PRP derivatives, such as platelet-rich fibrin (PRF), freeze-dried PRP, and iPSC derived platelets. The third generation, emphasis was on comparisons of PRP derivatives in terms of their ability to retain and release growth factors, mechanical strength, biodegradability, leukocyte population, and type. The fourth generation emphasized the incorporation of tissue engineering aspects in PRP therapy, for example, a combination of tissue-engineered periosteal sheets and PRP [11].

The article "Variability in Platelet-Rich Plasma Preparations Used in Regenerative Medicine: A Comparative Analysis" was published in 2022. Journal: Stem Cells Int.

We also need to consider the cost factor. There are broadly 3 types of methods available to prepare PRP: a completely commercialized large-scale production method, methods using commercial kits in small setups/clinics, and low cost/traditional methods for small clinics [3, 5, 12, 18]. A small setup may not want to introduce high-end robotics to process a few samples as dictated by patient load and public acceptance. From the point of view of personalized medicine, this brings us to the challenge of standardizing the available PRP processing procedure cost-effectively to ensure its wide-scale accessibility and usage (Figure 1).

Agencies like FDA (Food and Drug Administration) in USA, the Directive 2002/98/EC of the European Parliament and Council of January 27, 2003, and agencies in Japan have characterized and classified the PRP, laid down good manufacturing practices (cGMP) regulations and ensured compliance to guidelines [19]. PRP fits into the definition of minimally manipulated tissue and autologous blood product due to which it has avoided the regulatory hurdles of extensive preclinical and clinical trial testing, and as a result, its clinical practice may always outpace the supporting scientific data [1]. There are classification criteria determined by professional organizations available to help characterize and standardize the PRP/PRP products such as (1) PAW classification (2012), (2) Mishra's classification (2012), (3) PLRA classification (platelet, leucocyte, RBCs (red blood cells), and activation) (2015), (4) DEPA classification (dose of injected platelets, efficiency of production, purity of the PRP, and activation of the PRP) (2016), (5) MARSPILL classification (M: method; A: activation, R: red blood cells, S: spin, P: platelets, I: image guidance, L: leukocytes, L: light activation)(2017), (6) International Society on Thrombosis and Hemostasis (ISTH) classification (7) American Association of Orthopedic Surgeons (AAOS) edited consensus recommendations [2]. Parameters mentioned by these classifications are seldom used as they are expensive and time-consuming to implement. A center of excellence in regenerative medicine can do it [2].

We need to evolve from our long-standing understanding of pharmaceutical products where the pharmaceutical molecule works as a switch, turning on or off a particular pathway(s)/enzyme(s)/receptor(s). In the case of Biologics, the outcome is not determined by just one molecule but by a variety of factors simultaneously interacting at various levels. But first, the issue of standardization of PRP preparation involving standard protocols, equipment, and characterization of PRP/PRP-derived products needs to be addressed more broadly. The main objective of this study is to discuss the various procedures available to prepare the PRP and to investigate its efficacy.

The article "Variability in Platelet-Rich Plasma Preparations Used in Regenerative Medicine: A Comparative Analysis" was published in 2022. Journal: Stem Cells Int.

## 2. Materials and Methods

### 2.1. Search Strategy

This systematic review follows the protocol established by the Preferred Reporting Items for Systematic Reviews and Meta-Analyses (PRISMA) checklist. A comprehensive search was conducted in database search engines like EBSCOHOST, SCOPUS, and PUBMED. Prior to the literature search, the protocol was registered with the International Prospective Register of Systematic Reviews (PROSPERO ID: 307870).

### 2.2. Selection Criteria

Studies included in this systematic review met these inclusion criteria, (1) the research articles published between January 01, 2016, to July 31, 2022, and (2) articles with full texts and published in the English language. (3) Human studies conducted as prospective or Randomized Controlled Trial (RCT), (4) both in vitro and in vivo studies, and (5) articles describing the preparation methods for Platelet Rich Plasma (PRP).

### 2.3. Selection Strategy

A comprehensive literature search was conducted on July 31, 2022, using the electronic databases (PUBMED, EBSCOHost, and SCOPUS). Following search terms and keywords: ((“Platelet-rich plasma” OR “PRP” OR “Activated PRP” OR “Leukocyte rich PRP” or “Leukocyte poor PRP”) ^∗^ AND (“Regenerative Medicine” OR “Advanced Therapies” OR “Cell Therapy”)). Two authors (RVT and VJ) performed the literature search independently using the keywords for the articles to be included in this study. The selected articles were screened for any duplications following which, two reviewers (RVT & VJ) independently reviewed the title and abstract for further assessment of the studies for inclusion. The studies were excluded which did not address the study objective or meet the inclusion criteria. Finally, the full texts of the selected articles were examined to determine the final exclusion for our systematic review by reaching a consensus with all the authors involved. We also excluded articles which were editorials, opinions, commentaries, and book chapters. Any study which duplicated or involved the animal models was also excluded (Figure 2).

### 2.4. Data Collection & Analysis

After the content analysis of the selected articles, the following data were extracted from the study on a predetermined Excel sheet: (1) title, (2) type of study (“in vivo” vs “in vitro”), (3) product type, (4) PRP preparation procedure, (5) characterization of PRP, (6) additives or additional procedures used, (7) results.

The article "Variability in Platelet-Rich Plasma Preparations Used in Regenerative Medicine: A Comparative Analysis" was published in 2022. Journal: Stem Cells Int.

### 2.5. Quality Assessment

During the content analysis of the selected studies, the primary authors were contacted by email if the study did not provide the data needed for this study. We used the prevalidated Quality Assessment Tools for Observational Cohort and Cross-sectional Studies by the National Heart, Lung, and Blood Institute (NHLBI) (https://www.nhlbi.nih.gov/health-topics/study-quality-assessment-tools) to evaluate the quality of the selected study. In this systematic analysis, we regarded the study determined to be good and fair, worthy of being included in the resulting synthesis.

## 3. Results

### 3.1. Baseline Characteristics

We identified thirteen studies that reported the methods used in preparing PRP. All the studies considered were done in the last 5 years. Out of the 13 studies considered, twelve studies were in vitro studies, and one study was in vivo (Table 1). The final product of all the 13 studies considered was PRP with variations such as PRP releasate, Platelet lysate (PL), PR-SRGF (platelet releasate supernatant rich in growth factor), PRP gel, LR-PRP (leukocyte rich-PRP), LP-PRP (leukocyte poor-PRP), and UCB-PRP (umbilical cord blood-PRP). Venous blood was used to prepare the PRP in 12 research studies. However, there were differences in the method of collection. From the total 13 studies, in eight studies the blood was collected using commercial kits, of which two studies used a varying concentration of anticoagulants (sodium citrate) to study their effect on the yield of PRP, and one study used umbilical cord blood. The other six studies processed the collected blood with centrifugation using diverse types of centrifuges (horizontal or fixed angle rotors) and conditions (temperature or nontemperature controlled). One study used single centrifugation with variable *G* values [17]; three studies used double centrifugation with variable *G* values [9, 13, 18]; another study used single centrifugation while using a commercial kit [13]. All these methods followed pipetting to collect the PRP from centrifuged samples. Interestingly, the study by Bernardi et al. used a combination of apheresis with single centrifugation to collect PL and PR-SRGF [15]. Overall, four studies used apheresis as the direct method for preparing PRP. All the studies characterized the prepared PRP by looking at its comparative concentration of platelets in PRP and whole blood samples. All the studies used ELISA (enzyme-linked immunosorbent assay) method or kit method to measure the value of growth factors or other factors in PRP. Some studies measure specific factors such as IL-1Ra or lysophosphatidic acid, while others uses a panel ranging between 2-28 growth factors. Also, four studies considered the WBC population in the PRP sample. The PRP activation method was described in seven studies, and one of these study used freeze-thawing (FT) to activate PRP, two studies used FT with CaCl2 as an additional additive, another two studies used CaCl2, one study used CaCl2 with activated thrombin, and one study used activated serum with CaCl2. The efficacy of the PRP or PRP-derived product can be an indirect measure of the preparatory procedure. Six of the in vitro studies evaluated the efficacy of produced PRP on cell lines, two of these studies used commercial human cell lines, and one study used autologous stem cell lines. Overall, one study (in vivo) considered the efficacy of PRP and PRP gel on wound healing. Also, the study by Shimojo et al. analyzed the usage of PRP along with artificially engineered scaffolding for a sustained release of growth factors [11].

The article "Variability in Platelet-Rich Plasma Preparations Used in Regenerative Medicine: A Comparative Analysis" was published in 2022. Journal: Stem Cells Int.

## 4. Discussion

Commonly used procedures are as follows: venous blood collected using a vacutainer tube, syringe, or commercial kits are commonly used to prepare PRP [2]. Technologically advanced and equipped centers may use apheresis which gives leukocyte depleted PRP, which is a better quality PRP than venous blood derived PRP, which may have few leukocytes too [10]. However, there is a rising discussion about the presence of number and type of WBCs in PRP in some musculoskeletal studies, who argue that it is beneficial to have few WBCs in PRP [16], on the contrary, some others have stated that the leukocytes should be avoided in PRP preparations because of their potential proinflammatory effect [12]. Some centers worked with umbilical cord blood collection from the umbilical vein of the fresh placenta and added anticoagulants like acid citrate-dextrose (ACD) before further processing [20]. Large-scale production of PRP using closed systems in blood banks has been used [3]. Centrifugation is the main process used for density gradient-dependent separation of PRP from whole blood samples, unlike apheresis, or large-scale blood bank operations. Effect of normal temperature vs temperature-controlled, fixed angle vs horizontal rotors, single-spin method vs double spin methods, and use of anticoagulant on the fold of platelet yield/GF's is well documented [11, 21]. In cases of frozen PRP, the freeze-thaw cycle is considered to activate the PRP, as also the high-speed centrifugation (1000–10,000 G for the extended duration) and has been damaging to the platelets, causing degradation of platelets and release of platelet-derived factors [21]. The nonactivated PRP obtained from the previously mentioned methods is activated using Calcium chloride (CaCl2), fibrin and/or thrombin, and autologous serum to release growth factors (in vitro), both in case of fresh PRP and freeze-thawed PRP [11, 12, 14]. New engineering techniques such as biologic scaffoldings are also under analysis and development which would prolong the release of factors from platelets/PRP in vivo for sustained therapeutic effects [13].

The article "Variability in Platelet-Rich Plasma Preparations Used in Regenerative Medicine: A Comparative Analysis" was published in 2022. Journal: Stem Cells Int.

### 4.1. Addressing the Variability

#### 4.1.1. Procedure Variability

The PRP preparation procedures through generations of evolution have experimented with various physical parameters to progress towards the development of a standardized method and the most efficacious PPR/PRP product. The goal is still in distant sight. We lack complete and transparent large-scale data [1, 9]. The major reason for variations in the data and its comparability is due to variable approaches in preparation methodology such as the volume of blood collected for processing, method of collection (apheresis vs venous blood), source of sample (venous blood vs umbilical cord blood), different equipment, single centrifugation vs double centrifugation methods, normal temperature processing vs temperature-controlled settings, automation vs manual aspects, studies using fresh PRP vs Freeze-thawed PRP, usage of anticoagulants, and additives. [1]. Few authors believe that PRP products can be used without an activation agent because platelets are spontaneously activated upon exposure to dermal collagen and thrombin after in vivo injection [22, 23]. The usage of exogenous activating substances is controversial and required to explain the activation status since different PRP activation agents influence the physical form of the final product and may also influence the release curve of growth factors [2]. A study with 4 subjects, by Pulcini et al., [10] describe platelet yield by apheresis, measures selected platelet growth factors with respect to their osteogenic potential, and identifies the genes activated by the PRP components enhancing the osteogenic potential of cell lines used for in vitro study. The study by Ojea-P'erez et al. [3] describe the large-scale production (553 samples) of PRP. This study aptly describes the method of preparation of frozen PRP with monitoring of the quality/characteristics at regular intervals, showing almost no significant deterioration of quality/characteristics over time. Prior to using, the frozen PRP is thawed and activated using CaCl2, which will help in the release of factors from the platelets. The study supports its use in bone healing and regenerative medicine. A study by Ulasliet al. [21] recruited 12 subjects, talks about the collection of whole blood in sodium citrate (SC) 0.3% solution as an anticoagulant, which follows 3 different protocols, blood collection in tubes with 0.9 ml SC in protocol 1, 0.5 ml SC in protocol 2 and no SC in protocol 3. The PRP obtained from protocol 1 had high platelet count, highest TGF-b1 (transforming growth factor b1) and PDGF-BB levels, while protocol 3 had elevated levels of WBCs in PRP, correlating positively with the highest concentration of VEGF (vascular endothelial growth factor) and total VEGF levels (*p* < 0.001 for both and r:0.693, r:0.603, respectively). Another study by Machado et al. [18] recruited 32 subjects and used a remarkably simple, economical, and highly reproducible approach called Turn Down-Turn Up PRP Protocol Double Spin-Closed System, claiming results that are consistent with current standards of quality for PRP preparation for clinical trials suggested by the American Academy of Orthopedic Surgeons working group, who presented the MIBO statement. Their PRP preparation in a hospital facility is very economical, without considering the expenses of equipment and laboratory personnel. Another interesting study by Baba et al. [20] used Umbilical cord blood-derived PRP (UCB-PRP) from 9 healthy deliveries and compared its effect (osteogenic potential) on cryopreserved autologous Mesenchymal stem cells (MSC) derived from respective patients, after 3 years of storage. The study primarily considered secretion of 3 platelets derived factors platelet-derived growth factor-BB (PDGF-BB), an MSC proliferation accelerator, transforming growth factor *β*1 (TGF-*β*1) of TGF-*β* superfamily, an extracellular matrix production accelerator; and vascular endothelial growth factor (VEGF), an angiogenesis accelerator and measured the osteogenic potential of UCB-PRP, which was found to be intact even after 3 years of cryopreservation. The study did not investigate any adverse effects of cryopreservation on PRP or MSCs. A study by Darja Božič et al. observed variables like dimensions of the centrifuge rotor, volume of blood, and erythrocyte sedimentation rate affecting quality of PRP. It proposed a mathematically extrapolated model of obtaining enriched PRP and extracellular vesicles suspension by centrifugation after considering the variables. Its recommended procedure could manufacture a product high enough to merit the criteria for moderately concentrated PVRP by the PAW classification [9]. This study has numerous limitations.

The article "Variability in Platelet-Rich Plasma Preparations Used in Regenerative Medicine: A Comparative Analysis" was published in 2022. Journal: Stem Cells Int.

The observed studies had variations in procedures with very few similarities such as platelet yield and all of them measured and characterized GF. Even though their numerical data is available, statistical comparisons of these two parameters across different studies may be nonsignificant/difficult due to differences in their approach to getting platelet yield or the number and type of GF/platelet-derived factors considered.

#### 4.1.2. Patient Variability

Demographic variables like age, gender, presence, and absence of comorbidities, medication usage must be considered as they address the pathophysiological variations and hence the quality of PRP derived from the patients [24]. The in vitro study by Pulcini et al., [10] recruited 4 subjects between the age of 21 years and 59 years, none were on antiplatelet medications, and they studied the platelet yield and GFs in their samples. They applied the freeze-thaw cycles to activate platelets before using them to stimulate osteogenic growth in artificial human cell line cultures. The study notes variations in cytokines and GFs between aged and young subjects consistent with earlier studies [25]. Higher levels of GF's were noted in females and subjects <25 years of age. The study acknowledges reports from earlier studies where more proinflammatory cytokines were noted in the aged population in comparison to young subjects. However, it recommends considering larger sample sizes to draw more conclusions. Earlier studies have suggested that a higher concentration of cytokines and GFs had no relation to cell proliferation in cell lines used for testing PRP efficacy during in vitro studies [6, 26]. This raises an important question, what should be the ideal concentration of platelets, cytokines, and GFs to facilitate cell growth and proliferation in a particular tissue type. A study by Pulcini et al., [10] noted the effect of different dilutions of PRP on the proliferation of cells in commercial human cell lines. Another study by Velier et al., [5] used PRP/PRP gel in chronic wound care and addresses the patient related variability. The study compared 5 young healthy adults (median age 23 years) to 5 elderly patients (median age 85 years) with comorbidities like acute coronary syndrome, acute renal failure, stroke, obesity, hypertension, and diabetes, and on medications, with additional prescription for aspirin, clopidogrel, and fluindione. They found that the intensity expression of P-selectin after ADP stimulation was significantly higher in healthy donors compared to elderly (*p* = 0.03), while the basal expression of P-selectin showed no statistical difference. P-selectin expression is a measure of platelet activation [5]. Prothrombin concentration (*p* = 0.01) was measured higher in healthy donors. The researchers did not notice any significant difference in the biological characteristics of the therapeutic product PRP gel. The quality of the gel was correlated to the rate of formation. The faster the gel was formed, the more consistent it was. Linear correlations were found between biological parameters and PRP gel time formation. Overall, this study indicates that antithrombotic drugs have no impact on platelets functionality in PRP and PRP gel production. The limitations of the study were the small sample size, lack of evaluation on effects of oral anticoagulant therapy on PRP gel formation, and the PRP processing method had lower platelet yield in comparison to other recorded methods [5].

The article "Variability in Platelet-Rich Plasma Preparations Used in Regenerative Medicine: A Comparative Analysis" was published in 2022. Journal: Stem Cells Int.

#### 4.1.3. Characterization of PRP

The product derived following a standardized preparatory protocol requires desired measurable characteristics (Figure 3). This is an indirect measure of the potential of the preparatory procedure followed. The measurable characteristics will have to be in a range defined by different professional organizations [2]. The measurable characteristics of PRP (in comparison with whole blood/plasma measurements) are platelet count/folds of platelet concentration, levels of GFs, cytokines, chemokines, proinflammatory and anti-inflammatory factors, adhesion molecules, lysosomal enzymes, and extracellular vesicles. The PRP contains a diverse group of factors which collectively are responsible for the therapeutic outcomes [4] (Figure 4). But there are no studies available which consider the broader picture. This is due to the extensive nature of the parameters which need to be considered and the limitation of resources available for the process [2]. Different cell types and tissues have variable requirements of GFs or cytokines for their proliferation; also multiple of these factors can have overlapping functions in different cell types [4]. This highlights the need to consider the tissue specific requirements of the constituents in PRP/PRP products. The majority of the PRP studies have involved the musculoskeletal system and aesthetic medicine [1]. Most of the PRP preparation methods considered here can obtain higher platelet concentrations as compared to whole blood. These samples on stimulation or mixing with activators, can release various platelet factors which are the ultimate effectors of PRP therapy. Some studies have appreciated few WBCs in their PRP preparation. These studies claim that presence of certain types and number of WBCs in PRP may help in healing musculoskeletal injuries [2]. The activated PRP shows elevated levels of several factors, the composition of which has been characterized in several in vitro studies using standard ELISA based kits [3, 14, 15].

### 4.2. Outcome Measurements

#### 4.2.1. In Vitro Studies

Studies have measured platelet derived factors in PRP and were able to demonstrate specific proosteogenic gene activation in MSC derived commercial human cell lines [13, 18, 27] and umbilical cord derived human autologous MSC cell lines [20]. The product was characterized in terms of platelet yield and growth factors, proliferation of the MSC's in cell lines, and activation of specific genes was noted to measure the efficacy of the product.

The article "Variability in Platelet-Rich Plasma Preparations Used in Regenerative Medicine: A Comparative Analysis" was published in 2022. Journal: Stem Cells Int.

#### 4.2.2. In Vivo Studies

Study by Popescu et al. [2] used commercially available kits, all requiring blood collection and centrifugation, delivering injectable products which were divided into distinct groups and compared as (1) A-PRP (Activated PRP), (2) nonactivated PRP Vs calcium activated PRP, (3) human follicle mesenchymal stem cells plus A-PRP, (4) PRP plus Hyaluronic acid (HA) biofunctionalized scaffolding, and (5) PRP with fat graft and adipose derived MSC. Variations were seen in the quality of the product prepared using vacuum blood collection tubes with anticoagulant, anticoagulant prefilled syringes, and blood collection bags with anticoagulant. The product was characterized in terms of platelet yield and growth factors, activation of specific genes was noted, and clinical efficacy was the ultimate measure of the product's quality. Study by Velier et al. proved that the PRP's wound healing potential shows that it can be converted into gel form and applied as dressing. This emphasizes the efficacy of the PRP in treatment of chronic ulcers [5]. Musculoskeletal system-based studies have demonstrated safety and efficacy of PRP in human studies [1, 17]. We are now looking at the 4th generation approach where it is possible to design methods (using engineering techniques) to maintain slow and sustained release of platelet derived factors in vivo [13, 27].

When we discuss standardization of PRP preparation procedures, we must consider the commonality in the various reported PRP preparation procedures. The desired outcomes of PRP preparation are (1) high yield of platelets, (2) enhanced level of platelet derived factors in activated PRP, (3) sterility of the product, and (4) reproducibility. A 2013 study by Shwetha et al. [12] describe a simple and reproducible technique used to produce PRP from 22 different subjects. It reported the highest yield of platelets (8.8 to 9.3 folds after 2nd spin), more than by any study so far. The study uses 5 ml tubes containing 3.2% sodium citrate BD vacutainers with 0.5 ml SC anticoagulant, subjected to a double spin method at low speeds (300 g ×5 min 1st spin and 700 g×17 min 2nd spin) and variable temperature (12 degree C and 18 degree C). The temperature differences did not lead to any statistically significant platelet yield differences. The platelet pellets obtained after the 2nd spin were resuspended and activated using CaCl2 and/or thrombin. The sample was centrifuged at 3000 g to measure GF's and other platelet factors. The GF levels were variable in comparison to other previous studies, but it showed increased alpha granule release by calcium. Anti-inflammatory cytokines and chemokines showed no major differences between plasma and activated PRP. Proinflammatory cytokines are the ones that showed a significant increase in activated PRP. There are similar studies in the recent past claiming to develop high yield PRP. Therefore, we suggest that rather than focusing too much on various procedures for a good yield and irrespective of the procedures, we should focus on achieving a desired range of platelet yield, desired quality of PRP and desired level of platelet derived factors from that yield, in other words, getting a product which is enhanced in all parameters. The final product may be highly concentrated, in terms of constituents and can be diluted to desired proportions for its in vitro or in vivo or tissue specific application. The study by Pulcini et al. [10] points towards an interesting approach where serial dilutions of PRP can help us determine the optimum level of platelets and factors customized for a particular tissue or pathological condition. This approach finds support in the evidence found in a study conducted on 29 subjects by Cassano et al. [28] where bone marrow aspirate (BMA) was collected by the same surgeon. Each sample was divided and processed using two types of commercially available kits. PRP was processed using a standardized kit and method. The biologic autologous conditioned serum (ACS) was derived from it and used to evaluate the osteogenic potential of BMA derived stem cells, like in prior studies [7, 29]. Factors like IL-1ra, present in ACS, correlated positively with osteogenic activity [8, 28]. This study highlights usage of tissue specific requirements parameters to define quality of the PRP. This is in line with other musculoskeletal in vitro studies which have highlighted the effect of specific platelet derived factors on the osteogenic potential of stem cell lines [13, 18, 27]. A study involving 15 subjects by Bernardi et al., [15] also highlights that freeze-thawing technique for PRP can damage platelet membranes and may potentially affect the quality of PRP, especially in terms of slow and sustained release of factors in vivo. This could affect the clinical outcome of PRP. These findings can aid us in selecting between freshly prepared PRP and freeze thawed PRP for specific applications. For in vivo effects, the interaction of injected PRP and/or platelet derived factors with the local tissue depends on the characteristics of the product, and the altered pathophysiological parameters at the site of lesion. Some randomized studies have documented this interaction in osteoarthritis [8, 30]. More randomized studies are needed to understand the full scope of the nature of this interaction in different tissues as the requirements can be tissue specific [28, 31].

The article "Variability in Platelet-Rich Plasma Preparations Used in Regenerative Medicine: A Comparative Analysis" was published in 2022. Journal: Stem Cells Int.

### 4.3. Limitations

In this study we evaluated the different procedures utilized in preparing PRP, several factors like harvesting techniques, blood collection technique, presence or absence of activators, method of centrifugation may affect the composition of the PRP which were not compared due to lack of reporting of comparable data and resources. PRP has several applications which were beyond the scope of this article and so were not included. A different study for reviewing the multiple functions and utilizations of PRP can be performed. This study was limited to only in vitro and in vivo research in human models; animal studies were excluded from this research. Another limitation was lower human participation in few studies and the lack of uniformity in duration of the research performed.

## 5. Conclusion

Considering the variabilities in PRP preparation procedures, study by Machado et al. describes a simple, economical, highly reproducible approach and meets the current standards suggested by the American Academy of Orthopedic Surgeons working group, who presented the MIBO statement. Its platelet yield was 4.17-fold greater than the baseline platelet count. This study is an example of a systematic approach to attain the desired standardization in PRP preparation. Another study by Amable et al. describes a simple and reproducible technique to produce PRP, reporting 8.8-to-9.3-fold platelet yield. There is a clear relationship between the platelet yield and efficacy of the PRP/PRP product. A study by Sanchez et al. established that compared with hyaluronic acid injection in the osteoarthritic knee, PRP produced using the single spin technique, reaching 2-fold concentration, showed a superior effect [32]. This evidence suggests that even relatively low platelet concentrations may be effective. Interestingly, some studies have also noted that extremely high platelet concentrations (6-fold) may induce an inhibitory effect on osteoblast activity and healing processes [33]. Despite several recommendations, there is lack of consensus on the optimum concentration of platelets which is necessary to induce tissue repair. Therefore, a potential futuristic approach could be to obtain a highly concentrated product using either of the two above mentioned high yielding methods, which can be used in variable dilutions to obtain a tissue/pathology specific therapeutic desired level of platelets and activate. We recommend multicentric, randomized in vivo and in vitro studies to further evaluate the features of PRP derived factor pool, study their multidimensional interaction in vivo, and their rate of release, when using biologic scaffoldings. This will facilitate designing of enhanced therapeutic procedures/products. Careful consideration should be given to patient variability and tissue/pathology specific PRP production methods when formulating any universal guidelines.

The article "Variability in Platelet-Rich Plasma Preparations Used in Regenerative Medicine: A Comparative Analysis" was published in 2022. Journal: Stem Cells Int.

## Figures and Tables

**Figure 1:** Preparation of PRP.

**Figure 2:** The PRISMA protocol diagram for study selection.

**Figure 3:** Evaluation of PRP preparations.

**Figure 4:** PRP components and Function.

**Table 1:** Includes various methods used to prepare PRP. Includes type of study, preparation method, characterization of products, any additives used, and the results.

S. No	Articles	Type of study	Injectable product/product type used	PRP Preparation Method	Product Characterization	Additives used/ Additional procedures	Results
1	Apheresis Platelet Rich-Plasma for Regenerative Medicine: An In Vitro Study on Osteogenic Potential	In Vitro	PRP	Leukodepleted platelet-rich plasma (PRP) was collected by apheresis from four donors using an automated blood collection system (Mobile Collection System MCS+, Haemonetics Corp., Boston, MA, USA), according to the manufacturer's instructions. Acid Citrate, Dextrose Solution A (ACD-A) was used as an anticoagulant.	**1**.Platelet count, **2**. fibrinogen levels,**3**. 28 growth factors and 8 GF receptor concentration, **4**. Effect on in vitro proliferation, **5**. differentiation of osteoblast cells. Effects of different PRP dilutions (from 1% to 50%) on cell viability, growth, and differentiation.	Platelet activation is conducted by single and double freeze-thaw cycles.	Mean PLTs content in PRP samples 4.6-fold higher. Similar trends of GF in all 4 samples, their relative concentrations were different.

2	Implementation of a closed platelet-rich-plasma preparation method using the local blood bank infrastructure at the Principality of Asturias (Spain): back to basic method and a demographics perspective after 1 year.	In Vitro	PRP	Closed system PRP preparation method using the infrastructure of a certified blood bank. **1**.Extraction of 150mL blood. Transported in butanediol plates (constant temperature 20-24ºC). **2**.First centrifugation (425g, 5 min, acc6, no brake, 22oC), to separate plasma fraction containing platelets with a press Compomat G5 (Fresenius) into a new bag. **3**.Second centrifugation (1328g, 12 min, acc9, break 4, 22oC), to separate approximately 30mL of PRP into a new bag from the remaining platelet poor plasma. **4**.The PRP is allowed to rest for 4 hours and kept overnight agitating at room temperature. **5**.The PRP is then distributed into 3 pediatric transfusion bags (10 mL each). **6**.Aliquots are frozen at -40ºC to allow platelet lysis and cargo release and can be stored for 2 years. The PRP is distributed to the petitioner hospital on dry ice. **7**.The PRP is prepared within 24 hours of extraction and stored frozen, and the cold chain is maintained until its use.	They prepared 553 PRP units in 1 year. 1. The Multiplex Technology was used to measure concentration of several relevant growth factors like EGF, HGF, PDGF-BB, VEGF-A, VEGF-D, FGF-23. 2. PRP validation done by measuring WBC counts and platelet counts in whole blood and PRP across various samples.	Thawed PRP and using CaCl2.	Individual variations in platelet derived GFs were noted amongst donors and the concentration of factors amongst the three frozen aliquots derived from a single donor remained constant.

3	The effect of the anticoagulant on the cellular composition and growth factor content of platelet-rich plasma	In Vitro	Freshly prepared PRP	Single phlebotomists used T-Lab (T-Biotechnology, Bursa, Turkey) standard 0.9 ml 3.8% SC containing PRP tubes and PRP tubes without anticoagulants. Approximately 26 ml's of venous blood was obtained from each participant via 21G butterfly needle from antecubital vein, and the first 2 ml of blood was discarded to avoid platelet activation during blood collection. An additional 3 ml blood was collected from all volunteers for complete blood cell analysis. Two T-Lab swing rotor centrifuges were used for PRP preparation. PRP volumes obtained were recorded with the use of a 10- mL graduated pipette. The platelet, RBC, and WBC concentrations of the fresh PRP products from each protocol and whole blood were determined using hematology analyzer. **Protocol 1**: Approximately 7 ml blood was collected into the tubes prefilled with 0.9 ml SC, then, they were centrifuged at 1000 g for 5 min. **Protocol 2**: Approximately 8 ml blood was collected into the tubes without anticoagulant. Then, 0.5 ml SC was added. Immediately after blood collection, they were centrifuged at 1000 g for 5 min. **Protocol 3**: Approximately 8 ml blood was collected into the tubes without anticoagulant. The first 2 ml of blood were discarded to avoid early activation of the platelets. Immediately after blood collection, they were centrifuged at 1000 g for 5 min.	The PRP's were compared regarding cellular content (rbc, wbc, platelets), capture efficiency of platelets (CE), concentrations and total doses of fresh studied vascular endothelial growth factor (VEGF), platelet derived growth factor -BB, (PDGF-BB), transforming growth factor b1 (TGF-b1) levels.	No additives/activators	CE, total platelet count was highest in protocol 1. The white blood cells (WBC) and VEGF were highest in protocol 3. The highest total TGF-b1 and total PDGF levels were obtained with protocol 1, while the highest total VEGF levels were obtained with protocol 3.

4	An in vitro long-term study of cryopreserved umbilical cord blood-derived platelet-rich plasma containing growth factors —PDGF-BB, TGF-*β*, and VEGF	In Vitro	UCB-PRP cryopreserved for 3 years and thawed.	UCB was collected by puncturing the umbilical vein after the expulsion of the placenta. Immediately after collection, UCB was mixed with ACD-A (Terumo Co., Ltd., Tokyo, Japan) for anticoagulation. Subsequently, the mixture was centrifuged twice (2,400 rpm, 10 min; 3,600 rpm, 10 min) at 20 °C to obtain UCB-PRP and UCB-derived platelet-poor plasma. UCB-PRP was cryopreserved at −80 °C until the time of use. UCB-PRP, thawed at room temperature just before use, was randomly allocated to the experiments. Immediately after collection, the concentration rates of UCB and UCB-PRP per 1 mL of platelet count were calculated. The concentrations of growth factors (i.e., PDGF-BB, TGF-*β*1, and VEGF) which were contained in UCB at baseline, 3 months, and 3 years of cryopreservation, were determined quantitatively according to enzyme-linked immunosorbent assay.	1. Baseline, 3 months, and 3 years. 2. Measured PDGF-BB, TGF-*β*1, and VEGF) using ELISA. 3. Measured platelet concentration	No information on additives/Activators.	1.growth factors in cryopreserved UCB-PRP were markedly elevated compared to those found in UCB at baseline. 2.Cryopreserved UCB-PRP possibly and advantageously induced the osteoblastic differentiation of UC-MSCs.

5	Stabilization of porous chitosan improves the performance of its association with platelet-rich plasma as a composite scaffold.	In vitro	Activated PRP	1. Preparation according to Perez et al., whole blood (WB) was collected in 3.5 mL vacuum tubes (Vacuette®, Campinas, SP, Brazil) containing sodium citrate 3.2% (w/v) as an anticoagulant. 2. centrifuged in a Rotina 380R centrifuge (Hettich® Zentrifugen, Tuttlingen, Germany) at 100×g for 10 min at 25 °C. 3. The upper layer was collected as P-PRP. 4. Concentration of platelets, WBCs, and RBCs in WB and P-PRP was determined using the ABX Micros ES 60 hematology analyzer (HORIBA ABX Diagnostics, Montpellier, France). 5. Activated P-PRP (aP-PRP) prepared using autologous serum (Ser) and 10% (w/v) CaCl2 solution as agonists in the following proportions: agonist/P-PRP = 20% (v/v); Ser/CaCl2 volumetric ratio = 9. (Autologous serum was prepared by collecting 5 mL of WB in tubes without anticoagulant. After 30 min of clot formation, WB was centrifuged at 2000×g for 10 min).	The scaffolding was characterized by porosity, non-cytotoxic, pore size and young's modulus. PDGF-AB and TGF-*β*1 were measured using ELISA kits.	Autologous serum and CaCl2.	SPCHTs showed controlled release of the growth factors TGF-*β*1 and PDGF-AB. All the variations of stabilized scaffoldings showed cell differentiation more than non-stabilized ones.

6	Clinical-grade quality platelet-rich plasma releasate (PRP-R/ SRGF) from CaCl2-activated platelet concentrates promoted expansion of mesenchymal stromal cells.	In Vitro	PRP-R (platelet-rich plasma releasate) /SRGF (supernatant rich in growt factors)	1.Leucocyte-depleted platelet-rich plasma (PRP) was obtained by plasma platelet apheresis from healthy donors. 2.PRP was manipulated in aseptic conditions (validated clean room). 3.Platelet activation was performed in PRP by addition of CaCl2. 4.Supernatants of centrifuged samples (PRP-R/SRGF) were separated into aliquots and stored at -80°C without the addition of heparin. 5. Microbiology analysis was done to rule out bacterial or fungal contamination.	1. Platelet concentration not available. 2. PDGF-AA, PDGF-AB, PDGF-BB, TGF-b, FGF, EGF, IGF-1 and VEGF levels were measured by ELISA.	CaCl2 used for activation.	PRP-R/SRGF was more active than FBS to expand BM- and AT-derived MSCs. PRP-R/SRGF treatment did not affect the expression of typical MSCs surface markers, neither MSCs differentiation potential nor their capability to inhibit activated T-cell proliferation.

7	The Number of Platelets in Patient's Blood Influences the Mechanical and Morphological Properties of PRP-Clot and Lysophosphatidic Acid Quantity in PRP	In vitro	PRP	1. Venous blood from healthy male and female volunteers aged between 20 and 60 years; nonsmokers; and absence of chronic hematologic, neoplastic, and/or infectious diseases (HIV+, HCV+, and HBV+). 2.Samples of collected blood to obtain a platelet count. 3. Samples were then centrifuged at 2500 rpm for 8 min at 25 ◦C. 4. The PRP portion was removed as two fractions of equal volume: the more superficial one, called fraction 1 (PRP-F1), and the part nearest to the leukocyte fraction, called fraction 2 (PRP-F2). Platelet counting of PRP-F1 (F1) and PRP-F2 (F2) was performed before placing F2 into sterile vials and activating it according to Endoret® kit using 10% CaCl2 at 37 ◦C for 1 h to create the platelet concentrate (F2-clot). 5. Moreover, the in vitro activity of the PRP clots on proliferation and migration of osteoblast-like cells was assessed together with LPA quantification that was done on PRP-F1 (F1), PRP-F2 (F2), and Endoret®-activated PRP-F2 (F2-clots). Plasma concentrates (F2-clots) prepared from PRP from patients with low platelet number (group A) and PRP from patients with high platelet number (group B) were compared.	1. Platelet number 2. LPA was quantified before and after PRP fractioning and activation.	CaCl2 used for activation	There was significantly higher plasma level of LPA in patients with a higher platelet concentration (group B) in comparison to those in group A (p < 0.05). This different concentration was evidenced in PRP but not in the clots. Higher level of LPA in PRP from patients richer in platelets should be considered as responsible for the higher hOB activity in bone regeneration.

8	The production method affects the efficacy of platelet derivatives to expand mesenchymal stromal cells in vitro.	In Vitro	Platelet lysate and SRGF.	1. Platelet apheresis were collected from 15 donors, transferred to 50-ml tubes (Falcon, Corning MA, USA) and stored at −80 °C. After 2 cycles of freezing/thawing the aliquots were centrifuged at 1600×g for 15 min at room temperature and the supernatants were collected, pooled, filtered using a 70 *μ*m cell strainer (Falcon, Corning MA, USA) and finally stored at −20 °C until use. 2. Preparation of PR-SRGF: From the apheresis sample, platelet activation was performed by adding CaCl2 at the final concentration of 0.04 M and after incubation at 40 °C for approximately 60min until complete clot formation. Bags were centrifuged for 5 min at 2200×g and the SRGF collected and stored at −80 °C	1. Concentration of PDGF-AB, PDGF-AA, PDGF-BB, EGF, VEGF, FGF-basic, IGF-1, TGF-*β*1 were quantified by using ELISA Kits. 2. Platelet concentration.	Freeze/thawing & CaCl2.	The concentration of PDGF-AB, PDGF-AA, PDGF-BB in PR-SRGF resulted to be respectively 5.7×, 1.7× and 2.3× higher compared to PL. PR-SRGF promoted a higher BM-MSC proliferation rate compared to PL not altering BM-MSC phenotype. Colony forming efficiency of BM-MSC expanded in PR-SRGF showed a frequency of colonies significantly higher than cells expanded in PL. BM-MSC expanded in PL or PR-SRGF maintained their immunomodulatory properties against activated lymphocytes even if BM-MSC expanded in FBS performed significantly better.

9	Platelet-Rich Plasma Centrifugation Changes Leukocyte Ratios.	In Vitro	LR-PRP & LP-PRP	1. Gel-tube Method ~10cc of blood was spun at ~950g for ten minutes in a tube containing 1-2cc of a gel with a density slightly higher than platelets. The bottom 3cc of the plasma layer was removed as PRP. 2. Double-syringe Method ~15cc of blood in an ACP double syringe (Arthrex ACP Double-Syringe System; Arthrex Inc., Naples, FL, USA) was spun at 300g for five minutes and the plasma layer was withdrawn as PRP. 3.Machine Method 90-180cc of blood was placed into an Angel PRP machine (Angel® Concentrated Platelet Rich Plasma System; Arthrex Inc., Naples, Florida, USA) and processed with the setting set for a hematocrit of 4%. 4.Yellow-top Tube Method An ACD-A blood collection tube (BD Vacutainer ACD, catalog #364606; Becton-Dickinson, Franklin Lakes, NJ, USA) was filled with blood and spun at 1000g for ten minutes. The buffy coat and 1-2cc of the plasma layer just above it was extracted for PRP. 5.Single-syringe Method 15cc of blood was drawn into a syringe containing 1.5cc of sodium citrate solution and spun for ten minutes at 1000g. 0.6cc just below the buffy coat and 4cc above the buffy coat were removed as PRP.	1.Platelet count 2. Leukocytes and granulocytes numbers.	None	There is a significant shift, increase in lymphocyte percentage and decrease in granulocyte percentage is evident across PRP preparation methods

10	Bone marrow concentrate and platelet-rich plasma differ in cell distribution and interleukin 1 receptor antagonist protein concentration	In Vitro	PRP and BMC	1. Blood (25 mL) was drawn into a syringe holding 4 mL acid citrate dextrose (ACD). 2. Bone marrow was aspirated from the iliac crest into a 30-mL syringe holding 4 mL ACD. 1 mL was retained as the BMA sample for the study, and the rest was separated into two 60 mL samples and processed in two systems; Magellan® (BMC-A) (Arteriocyte Medical Systems Inc.) and SmartPrep® 2 (BMC-B; Harvest Technologies Corp., Plymouth, MA). All aspirations were performed by the same surgeon (JGK). All samples were processed within 24 h of collection.	1. Cellular concentrations of Platelets, rbc, wbc were assessed for all samples. 2.FGF-1, PDGF‑BB, VEGF, IL-1*β*, IL-6, IL-8, TNF*α*, IL-1ra, IFN-*γ*, TGF-*β*1, TGF-*β*2, 3 were measured using ELISA.	None	Colony-forming units were increased in both BMCs compared to BMA (p < 0.0001). Surface markers were consistent with MSCs. Platelet counts were not significantly different between BMC-A and PRP, but there were differences in leukocyte concentrations. TGF-*β*1 and PDGF were not different between BMC-A and PRP. IL1ra concentrations were greater (p = 0.0018) in BMC-A samples (13,432 pg/mL) than in PRP (588 pg./mL). The IL-1ra/IL-1*β* ratio in all BMC samples was above the value reported to inhibit IL-1*β*

11	Turn down - turn up: a simple and low-cost protocol for preparing platelet-rich plasma	In vitro	PRP	**Turn Down-Turn Up PRP Protocol - Double Spin - Closed System**: 1. Collect the desired volume (8.5 ml) of blood through peripheral venous access directly into a vacuum tube with acid citrate dextrose (ACD) (1.5 ml). 2. Equalize the remaining vacuum in the tube. 3. Centrifuge the tube at 200 _x0001_g for 15 minutes with the tube cap facing down. 4. Carefully remove the tube from the centrifuge and support the tube in the downward position without turning the tube. 5. Under aseptic conditions, aspirate 3.5 ml of the hematic layer through the rubber cap. 6. Turn the tube to an upright position (cap facing up). 7. Centrifuge the tube at 1600 _x0001_g for 10 minutes with the lid facing up. 8. Under aseptic conditions, aspirate 3.5 ml of the superior part of the material (platelet-poor plasma, PPP). 9. Aspirate the desired amount of PRP (1-2 ml) from the lower part of the tube.	1.Platelet concentration was measured in whole blood and PRP.	None	Four methods obtained concentrations of platelets that were 1.15-, 2.07-, 2.18-, and 3.19-fold, respectively. With the turn down-turn up technique, 4.17-fold (95% confidence interval (CI)

12	Production of platelet-rich plasma gel from elderly patients under antithrombotic drugs: Perspectives in chronic wounds care.	In Vivo	PRP and PRP gel	**PRP gel preparation** 1. Venous blood: The 20-ml anticoagulated syringe was transferred to the PRP tube while the 10-ml non anticoagulated blood was transferred into the PRAS® Gel tube to obtain serum containing autologous thrombin. 2. Centrifugation of both tubes was performed at 900G for 12 minutes. 3. Through luer lock connection, PRP and autologous thrombin were collected from each single tube. 4. One ml of PRP was kept for quality control including complete blood cell count, aggregometry and P-selectin expression. 5. Remaining PRP and autologous thrombin were mixed in an 8-cm diameter glass cupule with CaCl2 in the following way: PRP was first added in the glass cupule, followed by 0,5 ml of CaCl2 and mixed for 10 seconds. Then, autologous thrombin was added and mixed for 10 seconds. From there, time formation for the gel was assessed visually every 30 seconds until complete gel formation.	1.Platelet concentration 2. P-selectin expression 3.rbc, wbc concentration 4. Platelet aggregation in response to TRAP-6 5.Coagulation profile 6. Autologous Thrombin 7. Fibrinogen	1. Autologous thrombin and Cacl2.	1. No significant difference was observed in the volume, composition (quantity of platelets, leukocytes, and red blood cells) and functionality of platelets from PRP except a higher ADP-induced P-selectin expression in healthy donors compared with elderly patients. 2. Autologous thrombin characteristics were similar in the two groups. Concentrations of theoretical thrombin generated in the serum and in the gel were inversely correlated with the time of formation of PRP gel (r2 = 0.57, p = 0.012).

13	Enrichment of plasma in platelets and extracellular vesicles by the counterflow to erythrocyte settling.	In vivo	Platelet and EV rich plasma	Blood in the vacutainer is centrifuged at 300g for 5 min to obtain EPP (Erythrocyte poor plasma). This fraction is seperated and centrifuged again at 700 g for 17 minutes to obtain PVRP/PPP (Platelet & extravesicular rich plasma/Platelet poor plasma). Citrate as anticoagulant.	5 populations of particles were followed by Flowcytometry -- P1: attributed mainly to erythrocytes but containing also leukocytes, P2 and P2^∗^ (in larger and in smaller scale settings, respectively): attributed mainly to activated platelets and larger EVs, P3: subpopulation of particles with a weak side scattering signal, and Pa^∗^+Pb^∗^: attributed to smaller EVs and lipoproteins.	None	Study noted variations in the platelet concentration and EV's in the suspension which were related to sample handling, number of centrifugations,processing time, temperature, ESR, centrifugation pull and volume of blood.

The article "Variability in Platelet-Rich Plasma Preparations Used in Regenerative Medicine: A Comparative Analysis" was published in 2022. Journal: Stem Cells Int.

## Data Availability

The data generated during the research and analyses are not available publicly but are available on request and are stored at Mendeley Data. The supplemental files (quality assessment standards and MIBO statement) are available on Mendeley data. https://data.mendeley.com/datasets/nmvmp6wmnf/draft?a=ec8ad4fb-e86b-40cd-bb3c-148ac5d3d40e.

## Additional Points

Pre-print: A preprint of this article has been published on Research square [31].
